RETRACTED

# DNMT1-Mediated DNA Methylation Targets CDKN2B to Promote the Repair of Retinal Ganglion Cells in Streptozotocin-Induced Mongolian Gerbils during Diabetic Retinopathy

**DOI:** 10.1155/2022/9212116

**Published:** 2022-03-07

**Authors:** Xue Wang, Jinling Zhang, Yujie Liao, Yiping Jin, Xiaoyan Yu, Hong Li, Qi Yang, Xiaomei Li, Ranran Chen, Danping Wu, Haohao Zhu

**Affiliations:** Department of Ophthalmology, Shanghai Fifth People's Hospital, Fudan University, Shanghai 200240, China

## Abstract

**Objective:**

DNA methylation played a vital role in the progression of diabetic retinopathy. In this study, we aimed to explore the role of DNA cytosine-5-methyltransferase 1 (DNMT1) in the development of early diabetic retinopathy and its potential underlying mechanism.

**Methods:**

Eight-week-old healthy Mongolian gerbils were used to establish type 1 diabetes using streptozotocin (STZ). Alteration of weight, fasting blood glucose, density of RGCs (Tuj1-labeled), and H&E-stained retinal cross sections were applied to evaluate the diabetic retinopathy mouse model. The global DNA methylation level of the retina at different time points after STZ injection was measured using the global methylation assay. Western blot was used to detect the protein expression of DNMT1, DNA methyltransferase 3A (DNMT3A), and 3B (DNMT3B). Quantitative reverse transcription-polymerase chain reactions (qRT-PCR) and western blot were used to determine the expression of CDKN2B. Cell proliferation and cell cycle were evaluated by the MTS assay and flow cytometry.

**Results:**

STZ injection caused the increased global DNA methylation level, which reached a maximum at 6 weeks after injection. Moreover, STZ injection caused the damage of RGCs. At 6 weeks after STZ injection, the expression levels of DNMT1 and DNMT3B were significantly increased in the STZ group. DNMT1-induced DNA hypermethylation inhibited the expression of CDKN2B (a negative regulator of cell cycle). DNMT1-mediated DNA methylation facilitated RGC proliferation via regulating the expression of CDKN2B.

**Conclusion:**

DNMT1-mediated DNA methylation played an important role in STZ-induced diabetic retinopathy via modulating CDKN2B expression.

## 1. Introduction

Diabetes is well known as a chronic metabolic disease, which is characterized by hyperglycemia caused by the relative or absolute lack of insulin. Diabetes is divided into two most recognized types: type 1 diabetes (T1D) and type 2 diabetes (T2D). T1D is generally thought to be caused by an immune-associated destruction of insulin-producing pancreatic beta cells, while T2D is associated with insulin resistance and the lack of adequate secretion by the beta cells [1–3]. A variety of complications arises from chronic hyperglycemia, such as neuropathy, nephropathy, retinopathy, as well as cardiovascular disease [1]. Diabetic retinopathy is a common microvascular complication of diabetes, and affected a third of people with diabetes [4]. It was estimated that 40% people with T2D and 86% with T1D suffered from diabetic retinopathy.

RETRACTED

Diabetic retinopathy was recognized as a vascular disease, and the diabetic visual dysfunction might be caused by the vascular lesions. Increasing evidence convinced that retinal neuronal cells were also affected by diabetes [5]. Moreover, the damage of retinal neuronal cells caused by diabetes also resulted in the diabetic visual dysfunction. More importantly, retinal ganglion cell (RGCs) were wildly studied for the retinal neurons related to diabetes.^5^ It was reported that various animal models were used for exploring diabetes pathogenesis, such as Zucker Diabetic Fatty rats, BB rats, LEW 1AR1/-iddm rats, Goto-Kakizaki rats, and chemically induced diabetic rats.^1^ However, the diabetic animal models almost limited to mice and rats. The Mongolian gerbil is a diurnal rodent whose retinal structure is more analogous to that of human than of mouse [6]. Besides, the previous findings indicated that the retinal photoreceptors of Mongolian gerbils comprised 13% cones, while nocturnal mice and rats only possessed 1-3% [6].

Diabetic environment modulated the activities of enzymes related to epigenetic modifications, and some vital regulatory genes in the pathogenesis and progression of diabetic retinopathy underwent alterations of histone acetylation and methylation, as well as DNA methylation [7, 8]. DNA methylation was an important epigenetic mechanism for gene expression and genomic integrity [9]. These processes mainly rely on three different DNA methyltransferases: DNA cytosine-5-methyltransferase 1 (DNMT1), DNA methyltransferase 3A (DNMT3A), and 3B (DNMT3B). DNMTs methylate the C-5 ring position on the cytosine residues of enriched CpG dinucleotides in the promoter region of many genes [9]. In addition, DNMT1 was a vital enzyme to maintain DNA methylation, and DNA methylation was involved in diabetic retinopathy-associated many key genes transcriptional regulation [10, 11]. A number of studies indicated that enzyme-mediated DNA methylation affects cell proliferation, cell migration, cell differentiation, development, and aging [12–14]. Aberrant DNA methylation has been implicated in numerous human diseases, such as autoimmune diseases, neurodegenerative disorders, and cancer, as well as ocular diseases [15].

In this study, we established diabetic Mongolian gerbil model to explore whether DNA methylation participate in the protection of RGCs in diabetic retinopathy. Furthermore, we also explored the action of DNMT1 and its potential mechanism in the development of diabetic retinopathy.

RETRACTED

## 2. Materials and Methods

### 2.1. Streptozotocin- (STZ-) Induced T1D Model Establishment

The experiment was conducted under the approval of the Ethics Committee of Shanghai Fifth People's Hospital, Fudan University in strict accordance with the Guide for the Care and Use of Laboratory Animals published by the US National Institutes of Health. Healthy male Mongolian gerbils (8-week-old; *n* = 66) provided from the Zhejiang Academy of Medical Sciences (SCXK 2019-0002) were used in this study. All Mongolian gerbils were raised in the separate cages with free access to water and food, and maintained in a controlled environment (natural light at 26°C, relative humidity of 40%-70%, and noise less than 50 dB). A week later, Mongolian gerbils were divided into the STZ group (*n* = 33) and sodium citrate buffer injection (control) group (*n* = 33). The T1D models of Mongolian gerbils were established by intraperitoneal injection of STZ (150 mg/kg; Sigma, S0130, USA). STZ was dissolved in sodium citrate buffer (0.1 mol/L [pH 4.5], C1013, Solarbio, China). Random blood glucose was measured at 24, 48, and 72 h after injection. The model was successfully established when the blood glucose exceeded 16.7 mmol/L [16]. The control Mongolian gerbils were injected with the same volume of sodium citrate solution.

### 2.2. Cell Culture and Transfection

Well chamber slides were precoated with 100 mg/mL poly-D-lysine (A3890401, Thermo Scientific, Waltham, MA, USA) for 60 min and 20 mg/mL laminin (23017015, Thermo Scientific) for 30 min. After culling and ocular dissection, the retina of Mongolian gerbils was minced in 1.25 ml of papain (20 U/mL) (88285, Thermo Scientific) containing 50 mg/ml of DNase I (62.5 mL) and incubated for 90 min at 37°C. The retinal cell suspension was centrifuged at 300 g for 5 min and the pellet was re-suspended in 1.575 mL of Earle's balanced salt solution (14155063, Thermo Scientific) harboring 1.1 mg/mL of reconstituted albumin ovomucoid inhibitor (150 mL) and 56 mg/mL of DNase I (75 mL). After adding to the top of 2.5 mL of albumin ovomucoid inhibitor (10 mg/mL) to form a discontinuous density gradient, the retinal cell suspension was centrifuged at 70 g for 6 min and the cell pellet was resuspended in 1 mL of the supplemented Neurobasal-A (25 mL) (10888022, Thermo Scientific), 1× concentration of B27 supplement (17504044, Gibco), 0.5 mM of L-glutamine (A2916801, Gibco, GrandIsland, NY, USA) and 50 mg/mL gentamycin. The RGCs with a density of 125,000 cells/per well were seeded in an 8 well chamber slide and cultured in a humid incubator at 37°C supplied with 5% CO_2_ and 95% O_2_. Immunocytochemical staining of RGCs was performed using Tuj1 antibody (1 : 500, GB11139; Servicebio, Wuhan, China). Lipofectamine 2000 (Invitrogen, Carlsbad, CA, USA) was used for the transfection of siDNMT1 (5′-CACGAATTTCTGCAAACAGAAAT-3′) or siCDKN2B (5′-AACGGTTAACTGTAACGTTTTCT-3′) into RGCs.

RETRACTED

### 2.3. Retinal Histology Quantification

To evaluate the general retinal histology, the eyes of Mongolian gerbils were dipped into 1 mL FAX ocular fix buffer (Servicebio). Subsequently, paraffin embedding, sectioning, and hematoxylin and eosin (H&E) staining were performed. H&E-stained sections were imaged on a Nikon Eclipse Ti microscope with DS-Ri2 camera (Nikon Instruments, Melville, NY). Retinal thickness was measured using Nikon NIS-Elements software at 4 equidistant points along the outer retinal edge to either side of the optic nerve, where retinal thickness was defined as the length of a line orthogonal to the outer retinal edge and terminating at the inner retinal edge. Thickness was quantified using 6 technical replicates per animal and 3 biological replicates per genotype.

### 2.4. Global Methylation Assay

Genomic DNA was extracted with the DNeasy Blood & Tissue Kit (Qiagen, Hilden, Germany). Genomic DNA content was quantified by the Nanodrop One (Thermo Fisher Scientific). The global DNA methylation status was determined using the MethylFlash Global DNA Methylation ELISA Easy Kit (Epigentek, Farmingdale, NY, USA) according to the manufacturer's instructions. Briefly, 100 ng genomic DNA was added to each well. After washing, an aliquot of 5-methylcytosine (5-mC) detection complex solution was added and incubated at room temperature for 50 min. Then, the developer solution was added and the optical absorbance was measured with a microplate reader at 450 nm. The percentage of methylated DNA was calculated based on linear regression analysis.

### 2.5. Western Blot

Samples were homogenized in cold lysis buffer (1× phosphate-buffered saline pH 7.4, Thermo Fisher Scientific) containing protease inhibitor and phosphatase inhibitor cocktail (EMD Biosciences, La Jolla, CA). Protein concentration was determined using a Nanodrop ND-1000 spectrophotometer (Thermo Fisher Scientific). The samples were boiled for 5 min with loading buffer (39000, Thermo Scientific). Equal amounts of protein were separated on anykD mini-PROTEAN TGX polyacrylamide gels (Bio-Rad, Hercules, CA) and transferred to an Immobilon-FL PVDF membrane (Millipore, Burlington, MA). Then, the membranes were blocked with Odyssey blocking buffer (LI-COR Biosciences, Lincoln, NE) for 1 h at room temperature and then incubated with the primary antibodies including DNMT1 (1 : 2000; MA5-16169, Thermo Fisher Scientific), DNMT3A (1 : 500; MA5-16171, Thermo Fisher Scientific), DNMT3B (1 : 1000; MA5-38511, Thermo Fisher Scientific), CDKN2B (1 : 1000; MA1-12294, Thermo Fisher Scientific), and *β*-actin (1 : 1000; PA1-183, Thermo Fisher Scientific) overnight. Subsequently, the membranes were washed in 1× PBST and incubated with goat anti-rabbit Alexa Fluor 680 (1 : 5000; 35552, Thermo Fisher Scientific) or Goat anti-mouse IgG Alexa Fluor Plus 488 (1 : 2000; A32723, Thermo Fisher Scientific) for 1 h at room temperature. Finally, the membranes were subsequently imaged using an Odyssey Infrared Imaging System (LI-COR Biosciences).

RETRACTED

### 2.6. Quantitative Reverse Transcription-Polymerase Chain Reactions (qRT-PCR)

Total RNA was isolated using TRIzol reagent (Invitrogen). The concentration and purity of the RNA were detected with the use of nanodrop (ND-1000, Nanodrop Technologies). cDNA was synthesized with a RevertAid cDNA Synthesis Kit (Thermo Fisher Scientific). The primers designed with Primer Premier 5.0 software were synthesized by Beijing Tsingke Biological Technology (Beijing, China): CDKN2B: F 5′-CCCTGCCACCCTTACCAGA-3′, R 5′-CAGATACCTCGCAATGTCACG-3′; GAPDH: F 5′-TGGATTTGGACGCATTGGTC-3′, R 5′-TTTGCACTGGTACGTGTTGAT-3′. qPCR reactions were performed using Brilliant II SYBR Green qPCR master mix with low ROX (Agilent Technologies, Cedar Creek, TX) and monitored on a Stratagene Mx3000P cycler (Agilent Technologies).

### 2.7. Bisulfite Sequencing (BSP) PCR

The UCSC Genome Browser was used to explore the promoter sequences of Cdkn2b. BSP primers for the identified promoter sequences were drafted using MethPrimer software. Bisulfite conversion of genomic DNA extracted from the samples was performed using an EZ DNA Methylation-Gold Kit (ZYMO Research, Irvine, CA, USA). The bisulfite-treated DNA samples were then subjected to PCR amplification. PCR products were cloned using a ZeroBack Fast Ligation Kit (Tsingke, Beijing, China) and sequenced. Methylation of CpG sites was analyzed using the quantification tool for methylation analysis (QUMA).

### 2.8. Cell Proliferation Assay

Cell proliferation was determined by 3-(4,5-dimethylthiazol-2-yl)-5-(3-carboxy-methoxyphenyl)-2-(4-sulfophenyl)-2H-tetrazolim (MTS; Promega, Madison, WI, USA). After transfection, RGCs were treated with 20 *μ*L MTS and incubated for 1.5 h at 37°C. Finally, the absorbance was assessed at 490 nm using Varioskan Flash (Thermo Scientific).

### 2.9. Flow Cytometry

After transfection for 48 h, RGCs were collected, detached with 0.25% trypsin, and adjusted to a density of 1 × 10^6^ cells/mL. Then, the cell suspension (100 mL) was supplemented with 50 mg of PI solution (containing RNase) (40710ES03, Shanghai Qian Chen Bioscience & Technologies, Shanghai, China) for 30 min without light, and filtered with a 100-mesh nylon filter. Flow cytometry (Becton Dickinson, Franklin Lakes, NJ, USA) was used to record the cell cycle at 488 nm by red fluorescence. The experiment was conducted in triplicates.

RETRACTED

### 2.10. Statistical Analysis

Statistical analysis was conducted using the SPSS 21.0 statistical software (IBM, Armonk, NY, USA). All data were obtained from three independent experiments and subjected to normality test. The measurement data were presented as mean ± standard deviation. Comparisons between two groups were analyzed using a t test. Data conforming to normality among multiple groups were analyzed using one-way analysis of variance (ANOVA), followed by a Tukey post hoc test. The data with skewed distribution were analyzed using Dunn's multiple comparison post hoc test in the Kruskal-Wallis test. *P* < 0.05 was considered statistically significant.

## 3. Results

### 3.1. Generation and Validation of Diabetic Retinopathy in Mongolian Gerbils with Retinal Ganglion Cell Destruction

Multiple researches suggested that STZ was generally considered as the most effective diabetogenic chemical used in diabetes research [17]. STZ served as cytotoxic glucose analogues that tended to accumulate in pancreatic beta cells through glucose transporter 2, and ultimately led to DNA fragmentation. Therefore, we used STZ to establish diabetes models in Mongolian gerbils. After STZ injection, Mongolian gerbils in STZ group gradually presented diabetic symptoms of water intake, food-intake and urine volume increase. In addition, diabetic Mongolian gerbils became torpor, hunched, and fur-desiccated (Figure 1). Besides, some Mongolian gerbils in STZ group got cataract at 12 weeks after STZ injection (Figure 1). The related alteration of weight and fasting blood glucose were recorded in Table 1. Tuj1 antibody was used to recognize the nerve cells to evaluate the damage of RGCs. As shown in Figure 2(a), RGCs presented the most significant damage at 6 weeks after STZ injection. Meanwhile, after STZ injection for 6 weeks, retina was also markedly thinner than controls. Besides, STZ injection group exhibited the disrupted lamination and presentation of large-scale cell death in both inner and outer nuclear layers (Figure 2(b)). Further study found that diabetes-related retinal degeneration was most severe in the central area, with an average 45% reduction (but unaffected peripheral region) in Mongolian gerbils at 6 weeks after STZ injection (Figure 2(c)).

RETRACTED

### 3.2. DNMT-Mediated DNA Methylation Was Significantly Increased in the Early Diabetic Retinopathy

In order to clarify whether and when DNA methylation was involved in the process of diabetic retinopathy, we detected global DNA methylation in retina at 2, 4, 6, 8, 10, 12, and 14 weeks after sodium citrate buffer or STZ injection. The results showed that STZ injection increased the global DNA methylation level, which reached the maximum level at 6 weeks after injection; however, global DNA methylation level was decreased until it returned to the control level at 12 weeks after STZ injection (Figure 3(a)). On average, the global DNA methylation level in the retina of STZ-injected Mongolian gerbils was significantly higher than that in the control group (Figure 3(b)).

Since DNA methylation was catalyzed by methyltransferases (DNMTs proteins),^9^ we detected the expression level of DNMT1, DNMT3A and DNMT3B in the retina of Mongolian gerbils at 6 weeks after STZ injection. As shown in Figures 3(c)–3(d), compared with the control group, the expression levels of DNMT1 and DNMT3B in the STZ group were significantly increased, while the expression of DNMT3A was not changed.

### 3.3. DNA Hypermethylation Suppressed CDKN2B Expression in Mongolian Gerbils at 6 Weeks after STZ Injection

DNA methylation often occurred in the upstream regulatory regions of genes [18, 19]. CDKN2B was widely known as a negative regulator of cell cycle progression [18, 20]. Therefore, the expression levels of CDKN2B gene and its protein in RGCs were detected at 6 weeks after STZ injection, and the results revealed that the mRNA and protein expression of CDKN2B were significantly decreased after STZ injection (Figures 4(a)–4(c)).

In the six cpG-rich regions in the upstream regulatory region, methylation was detected by BSP and 25.9% of CPG sites were methylated in the control group and 74.1% in the STZ group (6 weeks) (Figure 4(d)). Significant CDKN2B hypermethylation spans from 1468 to 1299 nt were observed in the upstream regulatory region.

### 3.4. DNMT1-Mediated DNA Methylation Inhibited the Expression of CDKN2B and Facilitated RGC Proliferation

In order to verify the causal relationship of DNMT1 on CDKN2B methylation during diabetic retinopathy, siDNMT1 and siDNMT1+siCDKN2B were transfected into RGCs, and MTS and flow cytometry were used to test their effects on cell proliferation. DNMT1 knockdown caused a significant decrease of cell proliferation in RGCs (Figure 5(a)). Consistent with these results, the distribution of the S phase was increased by transfection of siDNMT1 in RGCs (Figure 5(b)). MTS also showed that the proliferation of RGCs transfected with siDNMT1+siCDKN2B was significantly increased compared with the siDNMT1 + NC group (Figure 5(c)). Similarly, the results of flow cytometry showed that the distribution of S phase cells was reduced in RGCs transfected with siDNMT1+siCDKN2B, while the distribution of G2 phase cells was increased (Figure 5(d)).

RETRACTED

## 4. Discussion

Diabetic retinopathy is a metabolic disease caused by long-term hyperglycaemia, and the pathogenesis and development of diabetic retinopathy are extremely complicated. The effects of diabetes on RGCs have been studied using some models, such as STZ-induced diabetes with disruption of the pancreatic *β* cells, Ins2Akita mice that spontaneously develop with type 1-like diabetes, and the spontaneously diabetic KKAY strain (a model of Type 2 diabetes). Barber et al. [21] found that 22 weeks of hyperglycaemia could lead to 23.4% reduction of the cell number in the retinal ganglion cell layer in Ins2Akita mice. Reduction in thickness of retina also has been detected in C57BL/6 mice with diabetes induced by STZ. STZ-induced diabetes in C57BL/6 mice could rapidly result in 20-25% fewer cells in the retinal ganglion cell layer after only 14 weeks of diabetes [22]. However, it was controversy about whether diabetes caused RGC death in C57BL/6 mice strain. Other investigators found no evidence of RGCs loss even after one year of diabetes using C57BL/6 strain [22–24]. In addition, a previous study revealed that diabetes might generate apoptosis of RGCs in KKAY mice [25]. In this research, our results demonstrated that STZ injection at 6 weeks could cause the significant damage of RGCs during hyperglycaemia in Mongolian gerbils, which might provide an important tool and means for further study on the pathogenesis and prevention of diabetic retinopathy.

Recently, the in-depth researches on the potential mechanism of DNA methylation in diabetic retinopathy were conducted, and the results demonstrated that diabetic retinopathy patients showed the higher global DNA methylation levels than that in diabetic patients without retinopathy, suggesting that global DNA methylation level might be a biomarker in diabetic retinopathy [26]. Consistent with this previous finding, our data showed that global DNA methylation was significantly enhanced in STZ-induced diabetic retinopathy in Mongolian gerbils. Additionally, DNA methylation was catalyzed by the DNMT family [9], which regulated DNA methylation to participate in cell proliferation, migration, and differentiation in healthy and various pathological conditions [27–30]. DNMT3B was proved to be necessary to establish de novo DNA methylation patterns during early development [31], while DNMT1 was primarily involved in maintaining methylation patterns that associated with DNA replication and cell proliferation [32]. A previous research reported that DNMT1-mediated MEG3 methylation contributed to endothelial-mesenchymal transition in diabetic retinopathy, thereby facilitating the progression of diabetic retinopathy [33]. This study found that DNMT1 was dramatically upregulated in RGCs of diabetic retinopathy, and DNMT1 modulated DNA methylation to be involved in diabetic retinopathy development.

RETRACTED

DNA hypermethylation was commonly found in the upstream regulatory regions of genes [18, 19]. Additionally, CDKN2B was proved to be a well-known negative regulator in cell cycle [18, 20]. Therefore, cell cycle was thought to be controlled by a dynamic balance between cyclin-dependent kinase (CDK) and CDKN, in which DNA methylation also played an important role [20, 34] In the present research, the results displayed that the expression of CDKN2B was markedly inhibited by STZ injection in Mongolian gerbils at 6 weeks. Moreover, significant CDKN2B hypermethylation was observed in the upstream regulatory region. These findings indicated that DNMT1-mediated DNA methylation to regulate the expression of CDKN2B in STZ-induced Mongolian gerbils. Based on the abovementioned findings, we speculated that DNMT1-mediated DNA methylation was involved in the progression of diabetic retinopathy through modulating CDKN2B. A recent study showed that DNMT1-mediated PPAR*α* methylation enhanced apoptosis of HRCPs and exacerbated damage of retinal tissues in diabetic retinopathy mice [35]. Thus, this study further verified the relationship between DNMT1 and CDKN2B in RGCs. Our results showed that DNMT1 knockdown promoted cell proliferation in RGCs, which was weakened by CDKN2B downregulation. In conclusion, DNMT1-mediated DNA methylation in the promoter region of CDKN2B gene inhibited the expression of CDKN2B, and ultimately accelerated the proliferation of RGCs. Overall, in the early stage of diabetic retinopathy, DNMT1-mediated DNA methylation in the promoter region of CDKN2B gene might play a protective role. However, after 6 weeks of STZ injection, the effects of DNMT1 gradually lost. Despite the limitation of DNMT1, these findings revealed a potential target for preventing the degradation of RGCs for diabetic retinopathy.

Diabetic retinopathy is now regarded as a neurovascular disease, which may cause severe vision impairment. Hence, to understand the early pathogenesis of diabetic retinopathy is crucial. Previous study has found that the synaptic function of rat retinas after 4 weeks of diabetes was decreased, for the low expression of presynaptic proteins. (Vis Neurosci. 2020 Sep 16; 37:E006. doi:10.1017/S095252382000005X.) Besides, David Sokolov et al. recently found that nuclear NAD + -biosynthetic enzyme NMNAT1 facilitates development and early survival of retinal neurons. (Elife. 2021; 10:e71185. Published 2021 Dec 8. doi:10.7554/eLife.71185) This study largely added to previous study of both early pathogenesis of diabetic retinopathy and early protection mechanism of RGCs.

RETRACTED

In conclusion, Mongolian gerbils might be a new animal model of diabetic retinopathy due to the faster degeneration reaction of RGCs. Besides, DNMT1-mediated DNA methylation regulated CDKN2B to promote RGCs repair in STZ-induced diabetic retinopathy.

## Figures and Tables

**Figure 1:** The appearance of Mongolian gerbils at various stages after sodium citrate buffer or STZ injection.

**Figure 2:** STZ injection caused the damage of RGCs. (a) Confocal images of retinal whole mounts showing Tuj1-labeled RGCs at 2, 4, and 6 weeks after STZ injection. (b) Representative H&E-stained retinal cross sections from sodium citrate buffer (SCB) and STZ injection groups at the indicated time. (c) The mean retinal thickness at the indicated time. ^∗^*P* < 0.05.

**Figure 3:** DNMT1-mediated DNA methylation was significantly increased in the early phase of diabetic retinopathy. (a) STZ injection upregulated the global DNA methylation level of the retina until 6 weeks after injection. (b) Quantification of the average 5-mC content in DNA methylation of the retina isolated from sodium citrate buffer injection (control) and STZ injection (STZ) groups. (c–d) Western blot showed the protein expression levels of DNMT1, DNMT3A, and DNMT3B. ^∗^*P* < 0.05, ^∗∗^*P* < 0.01.

**Figure 4:** DNA hypermethylation suppressed CDKN2B expression during diabetic retinopathy. (a) Quantitative analysis of CDKN2B mRNA expression in the control and STZ groups. (b) Western blot analysis was used to assess the protein levels of CDKN2B in the control and STZ groups. (c) Western blot analysis indicated the significantly decreased CDKN2B protein expression in the STZ group. (d) The position of the CpG sites at the upstream regulatory genomic locus of CDKN2B. Analysis of DNA methylation status at the upstream regulatory locus of the CDKN2B gene in control and WH groups determined by BSP. TSS: transcriptional start site. ^∗^*P* < 0.05, ^∗∗∗^*P* < 0.001.

**Figure 5:** DNMT1-mediated DNA methylation inhibited the expression of CDKN2B and facilitated RGC proliferation. (a) MTS assay was performed to compare the proliferation rates between NC (negative control) and DNMT1 siRNA-transfected RGCs. (b) RGCs were transfected with siDNMT1 or NC for 48 h and examined using flow cytometric analysis to determine the cell cycle phase distribution. (c) Quantification of the proliferation rates in siDNMT1+NC and siDNMT1+siCDKN2B-transfected RGCs using the MTS assay. (d) RGCs were cotransfected with siDNMT1+NC or siDNMT1+siCDKN2B for 48 h. Cells were analyzed by flow cytometry to determine the cell distribution at each phase of the cell cycle. ^∗^*P* < 0.05, ^∗∗∗^*P* < 0.001.

RETRACTED

**Table 1:** Weight and fasting blood glucose alteration after sodium citrate buffer injection and STZ injection.

	Time after injection	Weight (g)	Fasting blood glucose (mmol/L)
Untreated	—	75.66 ± 9.45	4.80 ± 0.79

Sodium citrate buffer injection	2 weeks	76.26 ± 10.01	4.43 ± 0.15
	4 weeks	77.33 ± 4.04	4.80 ± 0.62
	6 weeks	79.33 ± 9.45	5.33 ± 0.83

STZ injection	2 weeks	71.62 ± 1.15	28.13 ± 4.50
	4 weeks	66.64 ± 2.08	28.16 ± 1.45
	6 weeks	64.85 ± 2.64	29.05 ± 2.68

## Data Availability

The labeled dataset used to support the findings of this study are available from the corresponding author upon request.
